The article "Prehospital Emergency Service Use for Substance-Related Issues before and during COVID-19" was published in 2023. Journal: Emerg Med Int.

# Prehospital Emergency Service Use for Substance-Related Issues before and during COVID-19

**DOI:** 10.1155/2023/8886832

**Published:** 2023-04-17

**Authors:** Esra Kabadayi Sahin, Eren Usul

**Affiliations:** ^1^Department of Psychiatry, Ankara Yildirim Beyazit University Faculty of Medicine, Ankara, Turkey; ^2^Department of Emergency Medicine, Ankara Etlik City Hospital, Ankara, Turkey

## Abstract

**Objective:**

The COVID-19 pandemic disrupted the healthcare system and disproportionally affected individuals with substance use. This study aimed to evaluate the prehospital emergency medical service (EMS) use for substance-related health issues during the COVID-19 pandemic period and compare the changes with the pre-COVID-19 period.

**Methods:**

The prehospital EMS calls due to substance-related problems in overall Turkiye were analyzed retrospectively. The applications were categorized into the pre-COVID-19 period (May 11, 2019, to March 11, 2020) and the COVID-19 period (March 11, 2020, to January 4, 2021). These two periods were compared to if there were any changes in sociodemographic features of the applicants, the reason for EMS calls, and the dispatch results of the calls.

**Results:**

There were 6,191 calls in the pre-COVID-19 period and 4,758 calls in the COVID-19 period. According to the age groups, the number of applications of 18 years and under decreased, while the application of people 65 years and over increased during the COVID-19 period (*p* < 0.001). Considering the reasons for the EMS application, there was an increase in the calls due to suicide and transfers during the COVID-19 period. Besides, the EMS applications for court-ordered treatment decreased in the COVID-19 period (*p* < 0.001). There was no statistically significant difference in terms of dispatch results (*p* = 0.081).

**Conclusions:**

This study shows that the elderly group is at higher risk for substance-related medical problems. Suicide is an important risk among individuals with substance use. The increase in demand for ambulance transfer services can place a significant burden on prehospital emergency care. There is a need for measures to provide emergency and transport services, especially for the elderly and suicide attempts during any future case of emergency.

## 1. Introduction

As in the whole world, Turkiye has been struggling with the coronavirus disease 2019 (COVID-19) pandemic for more than two years. The pandemic has had significant psychosocial effects on society and brought major challenges to the healthcare system and public health policies [1, 2]. During the pandemic, the Emergency Medical Services (EMS) have been at the forefront of the fight against COVID-19. It has been reported that in the early stages of the pandemic, applications to emergency services decreased by up to 42% [3]. While this situation was related to the decrease in the application of some nonemergency cases, the fact that the delay of some important and urgent cases applying to health services may also have contributed to this situation. One of these important and urgent populations is the individuals with substance use.

The article "Prehospital Emergency Service Use for Substance-Related Issues before and during COVID-19" was published in 2023. Journal: Emerg Med Int.

The COVID-19 pandemic has disproportionately affected certain groups of people. Among the vulnerable populations are persons with alcohol or illicit substance use [4]. The stress, unemployment, decrease in social support, and lifestyle changes caused by the pandemic affected this sensitive group more severely and increased substance abuse [5]. Additionally, the high comorbidity rates of both physical and mental illnesses could lead to further health risks and complications for patients with substance use during the pandemic [6]. Moreover, alterations in the supply of the substances, increases in the costs, and decreases in the potency or purity of the drugs have changed the substance usage habits of the individuals and caused further medical problems [7].

Substance-related medical disorders and complications are highly frequent in EMS. It has been reported that emergency service admissions due to substance use vary in different periods of the pandemic. It has been stated that substance-related emergency service calls decreased in the initial stage of the pandemic, however, the applications increased after the stay-at-home order [8]. There is also some evidence that opioid overdose and deaths due to the overdose also increased during the pandemic [9, 10].

Although there is a limited number of studies on substance use-related emergency services admissions during the pandemic in the literature, it has been observed that most of these studies were conducted with a limited group of participants (limited to a certain city/state or a group of patients using a certain substance such as opioids) or limited for a short time. Therefore, we aimed to determine how the COVID-19 pandemic affected the pre-hospital emergency health services utilization due to all substance-related problems across Turkiye. Additionally, the study results also aimed to shed light on how problems related to substance use may affect prehospital health services use in case of a possible future disaster, and what precautions can be taken against these effects.

## 2. Methods

This study was designed as a retrospective observational study of country-wide substance-related EMS calls (1-1-2 ambulance call center) in Turkiye from May 11, 2019, to January 4, 2021. The first COVID-19 case was seen in Turkiye on March 11, 2020 [11] and was declared a pandemic on the same date by the World Health Organization (WHO). For this study, the pre-COVID-19 period was defined as May 11, 2019, to March 11, 2020. The COVID-19 period was defined as March 11, 2020, to January 4, 2021. Substance-related all EMS calls between the specified dates were derived from the Ministry of Health Department of Emergency Medical Services. From the deidentified data; age, gender, place of residence, the reason for EMS application, and dispatch result of those calls were recorded.

The article "Prehospital Emergency Service Use for Substance-Related Issues before and during COVID-19" was published in 2023. Journal: Emerg Med Int.

In order to determine substance-related calls, ICD-10 (International Classification of the Diseases-10) categories related to drug use were included (see: Appendix). The reasons for the EMS calls were gathered under six main categories (Table 1). The data was provided from either chief complaint recorded by the EMS call center or clinical impression recorded by the EMS provider. Cases whose electronic records could not be accessed or data were missing were excluded from the study (*n* = 952). Ethical approval for the study was granted by the local Ethics Committee of Dr Abdurrahman Yurtaslan Ankara Oncology Research and Training Hospital (date: June 22, 2022 no: 2022-06/1924).

### 2.1. Statistical Analysis

Data analysis was performed using IBM SPSS 25.0 (Armonk, NY: IBM Corp.) statistical package program. Kolmogorov–Smirnow test, skewness-kurtosis, and graphical methods (histogram, Q-Q Plot, Stem and Leaf, and Boxplot) were used to assess the distribution characteristics of the variables. The Pearson Chi-square (*χ*^2^) test was used to analyze categorical variables. Independent samples *t*-test was used for the evaluation of the quantitative data showing normal distribution. Descriptive data were reported as percentages, means, and standard deviations (sd). The statistical significance level was accepted as *p* < 0.05.

## 3. Results

There were 10,949 substance-related EMS calls included in the study. Of these calls, 56.5% (*n* = 6,191) were in pre-COVID-19 period and 43.5% (*n* = 4,758) were in COVID-19 period. The sociodemographic characteristics of the patients are given in Table 2 The mean age of patients who applied during the COVID-19 period was statistically significantly higher than in the pre-COVID-19 period (*p*<0.001). According to age groups, the number of applications of 18 years and under decreased, while the application of people 65 years and over increased during the COVID-19 period (*p* < 0.001).

There is no significant difference in patient gender or place of residence (*p* = 0.223 and *p* = 0.418, respectively). In the pre-COVID-19 period, males had a higher application rate to EMS than females which continued during the COVID-19 period. The number of EMS calls for both periods was almost five times higher within urban areas compared to rural areas.

The article "Prehospital Emergency Service Use for Substance-Related Issues before and during COVID-19" was published in 2023. Journal: Emerg Med Int.

Table 1 shows the reasons for EMS calls and the final result of their applications. When the reasons for EMS applications were compared between the two periods, there was an increase in the calls due to suicide and transport (transfers between health centers or hospital-to-home) during the COVID-19 period. Suicide attempt methods included self-harm with a firearm, sharp object, or jumping from height and poisoning with cocaine, opioids, psychostimulants, sedative hypnotics, and multiple substances or drugs. On the other hand, the EMS applications for court-ordered treatment decreased in the COVID-19 period (*p* < 0.001).

There was no statistically significant difference in terms of application results between the periods (*p*=0.081). The majority of the patients were transported to health care centers in both periods. The refusal of transport and on-site interventions slightly increased during the COVID-19 period; however, the differences between the two periods were not statistically significant (*p*=0.081).

When the substance-related EMS calls are evaluated according to Turkiye's seven geographic regions, the calls in the south and west regions (Mediterranean and Aegean regions) increased during the COVID-19 period, but the calls decreased in the Marmara region (*p* < 0.001). In the other four regions (Anatolia, East Anatolia, Southeastern Anatolia, and Black Sea regions), there was no statistically significant differences in the EMS calls between the two periods (Figure 1).

## 4. Discussion

This study showed that substance-related EMS calls were less in the COVID-19 period than in the pre-COVID-19 period. The age of the applicants seemed higher during the COVID-19 period and specifically elderly persons 65 years and over had a higher application rate. Applications to EMS for suicide attempts and transportations increased, while applications for court-ordered treatment decreased during the COVID-19 period. When compared according to geographical regions, while substance-related EMS applications increased in the southern and western parts of Turkiye, it was determined that the number of EMS calls decreased in the Marmara region.

It is shown that the prevalence of substance use at least once in their lifetime reaches 4.6% in Turkiye [12]. Although the rates of developing addiction vary, even a single use can cause substance-related health problems. Young age, male gender, low social support, living in an urban area, and having a comorbid psychiatric disorder are important risk factors for substance use [12, 13]. From this point of view, it is seen that EMS applications are high both in pre-COVID-19 and COVID-19 periods in males with high rates of substance use and those living in urban areas.

The article "Prehospital Emergency Service Use for Substance-Related Issues before and during COVID-19" was published in 2023. Journal: Emerg Med Int.

In our study, it was found that substance-related EMS searches after the pandemic decreased by approximately 23% compared to the prepandemic period. Studies have reported that applications to the emergency call service in the early stages of the pandemic generally decreased [14, 15]. It has been suggested that fear of infection and curfews may be effective in this. There are studies suggesting that it decreases or increases in the early period for substance-related applications, but their duration is quite limited [8, 9]. In a study covering the time of our study, it has been shown that EMS calls are generally decreased in Turkey [16]. Parallel to this, although it is seen that the number of substance-related calls has decreased, its percentage among the total calls is unknown.

In a study, emergency service visits decreased across all age groups, specifically in children and adults 65 years and over [17]. However, in our study, it was determined that the pandemic may have affected the age groups differently. While the substance-related EMS calls of 18 years and under decreased during the COVID-19 period, the application of people 65 years and over increased. There could be several possible reasons for this situation.

There are different results in the literature examining the effects of the pandemic on alcohol and substance use in children and adolescents. In some studies, it has been reported that cigarette and alcohol use decreased in this age group with the pandemic [18]. Contrary to this result, some studies showed an increased frequency of alcohol and cannabis use in adolescents [19]. The social isolation precautions might have resulted in less social pressure about substance use among adolescents and reduced substance use and so substance-related complications [20]. On the other hand, although the rates of substance use might not change, young people in this group might have applied to emergency services less frequently because they spent more time with their families or had difficulties in accessing health services.

It has been reported that the elderly group is affected more negatively by the pandemic than other age groups in different aspects. While current medical comorbidities and the impaired immune system may make older adults more vulnerable to medical complications [21], social isolation, fear of death, or insufficient social support may induce psychosocial distress in the elderly [22]. To cope with the increase in psychosocial stress, the frequency of alcohol and substance use may increase and this may cause exacerbation of chronic diseases. Additionally, older persons are more sensitive to any drug or substance side effects. Opioid analgesics or benzodiazepines given for the treatment of chronic pain or insomnia can cause many adverse effects in the elderly when used inappropriately. The elderly who could not go to the routine follow-up visits due to the changes in health services during the pandemic may have experienced these negative effects more frequently and therefore applied to the emergency services more frequently [23].

The article "Prehospital Emergency Service Use for Substance-Related Issues before and during COVID-19" was published in 2023. Journal: Emerg Med Int.

When the EMS application was compared according to seven geographical regions, substance-related EMS applications increased in the southern and western parts of the country, but decreased in the Marmara region, where the population density is high. It has been shown in other studies that there could be differences between the states in the frequency of EMS admissions [17]. Although more comprehensive studies should be conducted to elucidate the reasons for this situation, possible explanations for these differences may include the substance use profile of the population, the rate of COVID-19 cases, and the effects of pandemics on daily life and healthcare systems.

One of the most important outputs of this study is that the reasons for substance-related EMS calls have changed with the COVID-19 pandemic. Medical conditions were the most common reason for EMS admission in pre-COVID-19 and COVID-19 periods. This is a predictable outcome, as substance use-related complications and comorbid conditions are quite common [24]. Besides, our study also revealed that there was a significant increase in applications for suicide attempts during the pandemic period. It is known that suicide risk is higher in individuals with substance use than in the population [25]. Additionally, suicide attempts increased during the COVID-19 pandemic [26]. For this reason, it can be said that the negative effects of the pandemic on mental health are more pronounced in people with substance use and the dual risks increase suicide attempts in this group.

The transfers of the patients between healthcare centers and home-to-hospital also increased during the COVID-19 period. Transfers by ambulance have more than doubled. There may have been an increase in the number of patient transfers between health centers due to major changes in health services. As an example, some hospitals specifically cater to COVID-19-positive patients, while others care for a vulnerable patient group, such as cancer patients. The fact that people do not use public transportation or their vehicles due to restrictions may also play a role in this increase. In a study conducted in Turkiye, it was shown that there was an increase in the number of ambulance transport services from the hospital to the home during the pandemic [27]. This increase in the number of ambulance transfer services may indicate that it can create a burden for prehospital health services in case of future disasters.

The article "Prehospital Emergency Service Use for Substance-Related Issues before and during COVID-19" was published in 2023. Journal: Emerg Med Int.

On the other hand, EMS calls due to court-ordered treatment decreased during the COVID-19 period. This might be due to disruptions in legal screening and follow-up processes during the pandemic and the lockdown. It has been reported that there are some problems regarding these legal follow-ups for people with substance use during the pandemic in different countries [28].

Our results revealed that the dispatch results of the cases were not significantly changed during pandemics. Most of the cases were transported to the healthcare centers, and only a limited number of the cases refused the transportation. In previous studies, it has been shown that the refusal of transport to the hospitals has increased during the COVID-19 period [8, 9]. These different results can be explained by the fact that these studies were conducted in the relatively earlier stages of the pandemic and the fear of exposure to COVID-19 might be higher at that time in the community. At the time of our study, adaptation to living with the pandemic may have reduced avoidance behaviors.

Our study has several limitations. It has the limitations of a retrospective study. The design of the study is based on the collection of the electronic data from the EMS database; there could be possible misclassification of the cases or missing information. Since the causes of the suicide were not recorded clearly in every case, we could not discuss the reasons whether it was due to substance overdose or other suicide methods. Similarly, since the type of substance used by the individual was not recorded in each case, subgroup analyses related to substances could not be performed. On the other hand, this study is important as being a comprehensive study that evaluates all substance-related prehospital EMS applications across a large country.

## 5. Conclusion

In the pandemic, elderly patients with substance use may be specifically at higher risk for medical complications. The increased risk of suicide seen in the general population during the pandemic is also evident in substance users. The increase in demand for ambulance transfer services can cause a significant load on prehospital EMS. Prehospital emergency health services should take measures to meet the emergency response and transfer services, especially for elderly patients and suicide attempts in case of any future emergency states.

The article "Prehospital Emergency Service Use for Substance-Related Issues before and during COVID-19" was published in 2023. Journal: Emerg Med Int.

## Figures and Tables

**Figure 1:** Distribution of substance-related emergency health service calls by geographic regions during pre-COVID-19 and the COVID-19 period.

**Table 1:** Comparison of emergency health service application reasons and results between the periods.

		Pre-COVID-19 period (*n* = 6.172)	COVID-19 period (*n* = 4.742)	*p* ^*∗*^
Reason of application	Medical	3.551 (%57.5)^a^	2.613 (%55.1)^a^	**<0.001**
	Suicide	1.434 (%23.3)^a^	1.202 (%25.3)^b^	
	Others/Missing	906 (%14.6)^a^	538 (%11.3)^a^	
	Transfer	148 (%2.4)^a^	321 (%6.8)^b^	
	Trauma	89 (%1.5)^a^	64 (%1.3)^a^	
	Court-order treatment	44 (%0.7)^a^	3 (%0.1)^b^	

Result of application	Transported	5.590 (%90.6)	4.231 (%89.2)	0.081
	Refusal of transport	530 (%8.6)	469 (%9.9)	
	On-site intervention	43 (%0.7)	36 (%0.8)	
	Dead at scene	9 (%0.1)	6 (%0.1)	

^*∗*^: Pearson Chi-Square test. Each subscript letter denotes a subset of period categories whose column proportions do not differ significantly from each other at the 0.05 level. The bold *p* values are statistically significant.

**Table 2:** Characteristics of patients called emergency health services due to substance use.

	Pre-COVID-19 period (*n* = 6.172)	COVID-19 period (*n* = 4.742)	*p* value
Age (mean ± SD)	27.6 ± 11.5	29.0 ± 12.1	**<0.001** ^*∗*^
Gender (*n*, %)			
Female	2.009 (%32.6)	1.596 (%33.7)	0.223^+^
Male	4.163 (%67.4)	3.146 (%66.3)	
Residence (*n*, %)			
Urban	5.323 (%86.2)	4.064 (%85.7)	0.418^+^
Rural	849 (%13.8)	678 (%14.3)	
Age group (*n*, %)			
≤18 years	1.256 (%20.3)	770 (%16.2)	**<0.001** ^**+**^
19–64 years	4.872 (%78.9)	3.898 (%82.2)	
≥65 years	44 (%0.7)	74 (%1.6)	

^*∗*^Independent samples *t*-test, ^+^Pearson Chi-Square test. The bold *p* values are statistically significant.

## Data Availability

The data may be obtained from a third party and are not publicly available. Registry data may be available with permission of the Ministry of Health Department of Emergency Medical Services.

## Appendix

  ICD-10 diagnostic code list of complaints and dispatch reasons defined as substance-related calls
  Alcohol abuse (F10.1).
  Alcohol dependence (F10.2).
  Alcohol-related disorders (F10).
  Alcohol use, unspecified (F10.9).
  Cannabis abuse (marijuana) (F12.1).
  Cannabis dependence (F12.2).
  Cannabis-related disorders (F12).
  Cannabis use, unspecified (F12.9).
  Cocaine abuse (F14.1).
  Cocaine dependence (F14.2).
  Cocaine-related disorders (F14).
  Cocaine use, unspecified (F14.9).
  Hallucinogen abuse (F16.1).
  Hallucinogen dependence (F16.2).
  Hallucinogen-related disorders (F16).
  Hallucinogen use, unspecified (F16.9).
  Inhalant abuse (F18.1).
  Inhalant dependence (F18.2).
  Inhalant-related disorders (F18).
  Inhalant use, unspecified (F18.9).
  Opioid abuse (F11.1).
  Opioid dependence (F11.2).
  Opioid-related disorders (F11).
  Opioid use, unspecified (F11.9).
  Other psychoactive substance abuse (F19.1).
  Other psychoactive substance dependence (F19.2).
  Other psychoactive substance-related disorders (F19).
  Other psychoactive substance use, unspecified (F19.9).
  Other stimulant-related disorders (F15).
  Poisoning by, adverse effect of, and underdosing of cocaine (T40.5).
  Poisoning by, adverse effect of, and underdosing of diuretics and other and unspecified drugs, medicaments, and biological substances (T50).
  Poisoning by, adverse effect of, and underdosing of other and unspecified drugs, medicaments, and biological substances (T50.9).
  Poisoning by and adverse effect of heroine (T40.1).
  Poisoning by, adverse effect of, and underdosing of other opioids (F40.2).
  Poisoning by, adverse effect of, and underdosing of other and unspecified narcotics (T40.6).
  Poisoning by, adverse effect of, and underdosing of other and unspecified hallucinogens (T40.9).
  Sedative, hypnotic, or anxiolytic abuse (F13.1).
  Sedative, hypnotic, or anxiolytic-related disorders (F13).
  Sedative, hypnotic, or anxiolytic use, unspecified (F13.9).
  Substance use (Z72.2).
  Toxic effect of alcohol (T51).
